# Big Data-Enabled Analysis of Factors Affecting Patient Waiting Time in the Nephrology Department of a Large Tertiary Hospital

**DOI:** 10.1155/2021/5555029

**Published:** 2021-05-27

**Authors:** Jialing Li, Guiju Zhu, Li Luo, Wenwu Shen

**Affiliations:** ^1^School of Management, Hunan University of Technology and Business, Changsha 410205, China; ^2^Business School of Sichuan University, No. 24 South Section 1, Yihuan Road, Chengdu, China; ^3^Outpatient Department, West China Hospital, Sichuan University, Chengdu, Sichuan 610041, China

## Abstract

The length of waiting time has become an important indicator of the efficiency of medical services and the quality of medical care. Lengthy waiting times for patients will inevitably affect their mood and reduce satisfaction. For patients who are in urgent need of hospitalization, delayed admission often leads to exacerbation of the patient's condition and may threaten the patient's life. We gathered patients' information about outpatient visits and hospital admissions in the Nephrology Department of a large tertiary hospital in western China from January 1st, 2014, to December 31st, 2016, and we used big data-enabled analysis methods, including univariate analysis and multivariate linear regression models, to explore the factors affecting waiting time. We found that gender (*P*=0.048), the day of issuing the admission card (Saturday, *P*=0.028), the applied period for admission (*P* < 0.001), and the registration interval (*P* < 0.001) were positive influencing factors of patients' waiting time. Disease type (after kidney transplantation, *P* < 0.001), number of diagnoses (*P*=0.037), and the day of issuing the admission card (Sunday, *P*=0.001) were negative factors. A linear regression model built using these data performed well in the identification of factors affecting the waiting time of patients in the Nephrology Department. These results can be extended to other departments and could be valuable for improving patient satisfaction and hospital service quality by identifying the factors affecting waiting time.

## 1. Introduction

Long waiting times are recognized as a major obstacle to hospital care, affecting the quality of service and the establishment of friendly relationships with patients [1]. Due to the imbalance between the supply of and demand for medical resources, the problem of excessive waiting time is an issue for patients all over the world in outpatient, emergency, and hospitalization services. For patients, lengthy waiting time is not conducive to early treatment of their disease [2]. For hospitals, waiting time has an important influence on patient satisfaction [3]. Therefore, medical institutions committed to providing excellent service must effectively manage their clinic waiting times [4].

In some developed countries, the Emergency Department is the main channel for patient admission. For example, in the National University of Singapore Hospital, emergency patients account for more than 64% of all inpatients [5]. In China, outpatient clinics are the main channel by which patients enter the hospital. In the West China Hospital (WCH) of Sichuan University, outpatients account for about 67% of inpatients. The huge increase in demand for hospitalization in China has brought significant challenges to the management of hospital beds in medical and health institutions. In particular, large public hospitals with good equipment and technical conditions often have long waiting times. Due to the shortage of hospital beds, some public hospitals in China, such as the West China Hospital of Sichuan University, have an average of more than 6000 patients waiting in line every day. The waiting time for hospitalization of patients averages three months to six months, and some waits are more than one year [6].

Both the Emergency Department and the Outpatient Department receive inpatients. Inpatients generally require more services than outpatients, given the complexity of their diseases, so their waiting time is important. Therefore, in this study, we focused on factor analysis of the waiting time of admitted patients. To a certain extent, the hospitalization waiting time reflects the hospital's admission and discharge management level and the hospital's inpatient service quality [7]. Shortening the patient's admission waiting time will help improve the patient's admission experience and reduce the occurrence of medical disputes [8].

Different hospital departments have different admission characteristics, and the waiting time varies greatly in different departments. Therefore, under the advice of the administrator of the Admission Service Center, we chose the Department of Nephrology as the subject for the analysis of factors affecting the admission of patients, rather than discussing the determinants of inpatient waiting time for the entire hospital. This approach allows us to generate more specific, personalized admission management recommendations.

Several studies have demonstrated that long waiting times have negative impacts on the hospital's quality of service [9], patient satisfaction [10, 11], and hospital reputation [12]. Susanto and Chalidyanto [13] investigated waiting time and patient satisfaction in the pharmacy, using a cross-sectional study. Given the impact of waiting time on hospitals and patients, hospitals should take active measures to effectively manage the waiting times of patients.

There have been many studies into waiting time in healthcare institutions, focusing mainly on outpatients [14, 15] and Emergency Departments [16, 17]. The research has mostly been carried out from the perspective of the country, the region, or the entire hospital [18, 19]. For example, Geta and Edessa [20] investigated the factors affecting the waiting time of outpatients, using a questionnaire. Isfahani and colleagues [21] assessed the effects of a discharge lounge on decreasing patient waiting time and Emergency Department overcrowding, using a computer simulation. They found that the main factors leading to long patient waiting times are hindrances in patient flow and the occupation of Emergency Department beds by nonemergency patients. There have been relatively few studies into the waiting time of inpatients, and there is a lack of evidence-based management recommendations for hospitals.

Some research has focused on exploring which factors tend to increase the waiting time, including the overcrowding of patients, lack of healthcare providers, employee attitudes, work processes, length of hospital stay, and management problems [22–26]. However, this research primarily uses traditional methods, such as questionnaires, interviews [27], qualitative descriptions [28], and simulations [29]. For example, Aburayya et al. [30] collected questionnaires from 12 healthcare centers in the Emirate of Dubai in the UAE and found that the main causes of waiting time were high staff workloads, insufficient work procedures, employee-supervisor interaction problems, and lack of adequate facilities.

Data-driven methods are rarely used to explore the factors that affect the waiting times of inpatients. Data mining technology and machine learning methods have been successfully applied in many fields, such as intelligent diagnosis and treatment [31–33], engineering [34], and security [35]. The wide range of these applications suggests that data mining technology may be used to analyze the factors that affect waiting time. Multivariate linear regression analysis, using statistical significance to identify explanatory variables, has been suggested as an effective method for evaluation, using big data [36].

In this study, we addressed this issue. We used the Department of Nephrology, WCH of Sichuan University, as an example, and analyzed the data from admitted patients, using multivariate linear regression, a machine learning algorithm, to unearth the key factors affecting the waiting time of inpatients. We used these data to provide evidence-based suggestions for reducing waiting times.

The remainder of this paper is structured as follows. Materials and methodology are introduced in Section 2. Results obtained using linear models are presented in Section 3. The analysis of the factors is presented in Section 4. In Section 5, we provide a brief conclusion.

## 2. Materials and Methods

### 2.1. Study Setting

West China Hospital is a large tertiary hospital in western China. It is faced with an admission problem common to large hospitals: bed resources cannot meet the demand for admission, and patients usually wait a long time before admission. In response to the increasing demand for hospitalization, an Admission Service Center was established in 2013 to centrally manage hospital beds. The data for this study came from the registration system of the Admission Service Center.

To better understand the waiting time of inpatients, we first provide a brief overview of the admission process for inpatients of WCH.  Figure 1 is a schematic of the admission process.

#### 2.1.1. Outpatient Service

First, each elective patient needs to see a doctor in the Outpatients Department. The outpatient doctors then provide a patient admission card, according to the severity of their illness. An admission card is an important certificate for hospitalization. Patients without an admission card will leave the hospital.

#### 2.1.2. Admission Service Center

When a patient receives an admission card, they go to the Admission Service Center (ASC) to complete the hospital registration with information such as demographics, disease type, and insurance. After registration, a patient is added to the waiting list, sorted by registration date. A professional selects the patients who most need hospitalization services from the waiting list, based on their registration information. When a patient is selected, the professional will call the patient to ask if they have time to come to the hospital the next morning. Admitted patients who are notified by telephone and agree to hospitalization can go to the ASC to complete other procedures such as preoperative examinations, CT scans, and other diagnostic tests. The patient is conveyed to the ward at the appointed time.

#### 2.1.3. Discharge

Patients accept hospitalized services (including preoperative tests, treatment, and postoperative tests) and are finally discharged from the hospital after recovery.

Using this process, we defined the waiting time of inpatients as the time between the issuing of the patient's admission certificate by the outpatient doctor and the patient's formal admission for treatment.

### 2.2. Data Source

We first collected all of the data generated by the patients before admission from the Admission Service Center. The data included gender, age, date of application for admission (year, month, day, hour, and minute), registration date, outpatient diagnostic information, and subspecialty information. This information is the main resource used by medical staff when judging whether a patient is admitted to the hospital.

We extracted the admission data from the Department of Nephrology, West China Hospital, from January 1, 2014, to December 31, 2016. After deleting missing values and outliers, a total of 13,336 samples were obtained. All data were anonymized.

### 2.3. Data Preprocessing

After extracting the required fields, the data were preprocessed. We performed feature engineering on the original data to extract features for use in the model. The process of data processing is as follows.

First, males were coded as 1 and females as 2. Age was divided into four categories: juvenile (0–17 years old) as 1, young (18–40 years old) as 2, middle-aged (41–65 years old) as 3, and old (over 66 years old) as 4.

We then derived new fields based on the current fields. (1) Registration interval (RI) refers to the interval between the registration date and the date of issue of the admission card. (2) Standardized date of admission was split into two fields: the week of issuing the admission card (WIAC) and the applied period for admission (APA). We divided the latter into two periods: morning and afternoon. We labeled the weekday from 1 (Monday) to 7 (Sunday), and the applied period for admission was coded as 1 (morning) or 2 (afternoon). For example, a patient who had an admission card issued at 8 : 23 am on November 29, 2016, was coded as being issued with an admission card on Tuesday (assigned as 3) morning (assigned as 1). (3) Since many patients register on the same day after receiving the admission card, the week of the admission card date is very similar to that of the registration date. In the end, only the week of the admission card date was retained. (4) The outpatient diagnosis information was the outpatient doctor's record of the patient's condition. A new field, the number of disease diagnoses, was derived by counting the number of diagnosed items.

The seven independent variables used in this study are shown in Table 1. We divided the following independent variables into three categories. The first category was descriptive statistical information, including gender and age. The second category was time information, which contains three variables: WIAC, APA, and RI. The third category was disease information, including two variables, TD and NDD. TD was divided into five subgroups: vascular access, renal biopsy, peritoneal dialysis, after kidney transplantation, and others. NDD was divided into four levels. In the outpatient diagnosis field, the diagnosis of only one disease was assigned a value of 1, diagnosis of two diseases was assigned 2, diagnosis of three diseases was assigned 3, and four or more diseases are assigned 4.

### 2.4. Methods

After sorting and converting the original data, *R* software was used for data analysis and modeling [37]. We first summarized the data. The measurement data was described by the mean, and the counting data was described by percentage.

We then carried out a univariate analysis. The difference in the waiting time of inpatients between each group was analyzed using univariate analysis [38], and the relationship between continuous variables and the waiting time of inpatients was analyzed using the Spearman correlation [39].

Finally, we constructed a multivariate linear regression model to explore the factors affecting the waiting time of patients registered in the Nephrology Department. We used the fields in Table 1 as independent variables and waiting time as the dependent variable. We used stepwise regression to filter the independent variables. Variables with  *P* < 0.05 were selected as independent variables, at an inspection level of *α* = 0.05. The generalized variance inflation factor (VIF) and variance inflation factor were used to test the multivariate collinearity of the model. We assumed that there was no collinearity when GVIF or VIF was less than 2 [40].

## 3. Results

### 3.1. Descriptive Analysis

The descriptive analysis of the variables and sample information is shown in Figures 2–4.  Figure 2 is a descriptive analysis diagram of the variables age and gender. The dataset included 7,106 male patients, with an average waiting time of 5,72 days, and 6,230 female patients, with an average waiting time of 4.88 days. The number of male patients was slightly higher than that of female patients, and there was an approximately one-day gap in the average waiting time. The proportion of patients aged 41–65 was the largest, accounting for 46.75%. Middle-aged patients had the longest average waiting time, as high as 5.7 days.

Figure 3 shows an analysis of the time-related variables. During the admission period, we found that 56.46% of patients were registered in the morning (00 : 00–11 : 59), and 43.54% were registered in the afternoon (12 : 00–23 : 59). For the admission card, the number of patients on weekdays was much higher than that on weekends. Monday and Wednesday had the largest number of patients at 3,161 and 2,785, respectively. However, the waiting time on weekends was much higher than that on weekdays.

The characteristics of disease-related information are presented in Figure 4. In the Nephrology Department, TD is subdivided into five subspecialties. The proportion of cases of renal biopsy is the largest (33.05%), followed by vascular access (26.9%). The longest waiting time was for the peritoneal dialysis subspecialty (6.97 days). Most patients (78.43%) had only one diagnosis, and the corresponding average waiting time was relatively long (5.34 days).

The average registration interval was 1.46 days. This observation indicates that some patients did not register for hospitalization immediately after receiving the admission card. The average waiting time for patients admitted to the Department of Nephrology was 5.33 days, and the standard deviation was 22.17 days. The high value of the standard deviation was due to the fact that some patients have milder disease, and the hospital always prioritizes the admission of severe cases, leaving some patients waiting for a long time.

We used univariate analysis and multivariate analysis to examine which factors affected the waiting time of inpatients, and how the data reflected the problems delaying the admission of patients.

### 3.2. Univariate Analysis

This section describes a univariate analysis of the factors affecting the waiting time of patients in the Nephrology Department. The results are shown in Table 2. Gender, week of issuing the admission card, and disease type had statistically significant effects on patient waiting time (*P*<0.05). We then analyzed the correlation between the registration interval and the waiting time for admission. The waiting time of inpatients in the Nephrology Department was positively correlated with registration interval (*P*<0.01).

### 3.3. Multivariate Linear Regression Analysis

Taking the natural logarithm of waiting time as the dependent variable, we used stepwise regression to filter the independent variables. The week of admission, disease type, and the number of disease diagnoses were included in the model as dummy variables. The model results are as follows.

We used the coefficient of determination*R*^2^ to measure the goodness of fit of the linear model. We saw an *R*^2^ = 0.527, which shows that the regression line fits the observations well. For the model, we found *P* < 0.001, indicating that at a test level of *α* = 0.05, the fit of the multivariate linear regression equation can be considered to be statistically significant.

The results of the multivariate linear regression analysis are shown in Table 3. We found that all variables except age were statistically significant.

Gender (male, *P* = 0.048), WIAC (Saturday, *P* = 0.028), APA (PM, *P* < 0.001), and RI (*P* < 0.001) were the positive factors influencing the waiting time. Taking the RI as an example, the unstandardized coefficient *B*was 0.789, and the 95% CI was (0.712, 0.736), indicating that when the other factors remained unchanged, for every additional day of the registration interval, the waiting time increased by 0.789 days.

The WIAC (Sunday, *P* = 0.001), DT (after renal transplant, *P* < 0.001), and NDD (Four or more diseases, *P* = 0.037) were negative factors. Taking the DT as an example, the coefficient *B*of type four, after renal transplant was -3.091, which can be explained as follows: compared with type five, under the same conditions, the waiting time was reduced by 3.091 days for patients with the after renal transplant.

We performed a collinearity analysis on the above six statistically significant variables (Table 4). It can be seen that *GVIF* < 2and *VIF* < 2, which means that there was no collinearity in the independent variables in our model.

The significance of the standardized regression coefficients*β* was to compare the importance of different independent variables to the dependent variable by standardizing *B*. The importance of each factor to the waiting time can be compared according to the absolute value of the standardized regression coefficient of linear regression. The results showed that RI (0.724), WIAC (Sunday, 0.191), DT (after renal transplant, 0.139), NDD (≥4 diagnoses, 0.097), and WIAC (Saturday, 0.077) were the top five factors that had the greatest impact on the waiting time for admission (Figure 5).

## 4. Discussion

This study was based on data provided by the information platform of the Admission Service Center and used data mining technology to assess the determinants of inpatients' waiting time in the Nephrology Department of a tertiary hospital in western China. Based on the theoretical results presented in Section 3, we conducted interviews with the hospital's managers to learn more about the possible reasons behind the theoretical results. Finally, combined with observation of the actual situation of the hospital, we provide a theoretical basis for hospital administrators to take measures to shorten the waiting time for patients to be admitted to the hospital and improve the patient's admission experience.

### 4.1. Descriptive Information

This model showed that age had little effect on patients' admission, while gender was statistically significant. The waiting time of males admitted to the Department of Nephrology was 0.5 days longer than that of females. This is because there were more male than female outpatients (Table 2). Because Chinese hospitals require that men and women are not housed in the same ward, when the total number of beds is limited, higher numbers of outpatient visits for male patients lead to greater opportunity costs of waiting for beds, and the waiting time increases. This finding indicates that hospitals should adjust the ratio of male and female bed resource allocations and appropriately increase the number of admissions of male patients to meet different needs due to gender differences.

### 4.2. Time Information

The WIAC, RI, and APA had a considerable impact on the waiting time of patients. In general, patients who were issued an admission card on Sunday had shorter waiting times than those who were issued an admission card on Friday.

This result is related to the way in which the hospital is run and the resulting temporary release of hospital beds. The poor management of planned discharge from the clinical department of the hospital on weekends has led to the temporary discharge of some patients, and the Admissions Center has fewer staff on duty. After a patient is temporarily discharged, the hospital will admit patients who were issued an admission card and registered on-site on the same day. Therefore, patients who are issued an admission certificate on Sunday have shorter waiting times than those given a certificate on Friday.

From the perspective of the process of patient admission, the waiting time can be subdivided into indirect waiting time (the time between issuance of an admission card and registration at the Admission Center) and direct waiting time (the time between patients officially entering the waiting queue after registration and hospitalization). The registration interval reflects the urgency of admission, to a certain extent. The earlier a patient registers, the earlier he enters the hospital waiting system, and the shorter the direct waiting time. The length of the registration interval will directly affect the patient's waiting time for admission. Large hospitals should pay attention to the outpatient guidance service and guide patients to register effectively to reduce unnecessary waiting times.

Patients issued with admission permits in the afternoon wait longer. One possible reason is that the hospital releases fewer beds in the afternoon. According to the current operating rules of the hospital, the peak of admission and discharge is concentrated at 09 : 00–11 : 00 in the morning, lengthening the direct waiting time.

The hospital should strengthen the management of planned discharge. A reminder function can be added to the prehospitalization information system to remind patients of the admission progress through means such as SMS alerts, or telephone follow-ups, to realize the whole-process tracking of patients' medical treatment, improve service quality, and improve the medical experience.

### 4.3. Disease Information

This study shows that disease type 4 (after renal transplant) had a shorter waiting time for admission than other disease types. This is because in patients with a after renal transplant, taking immunosuppressants leads to a decrease in immunity, resulting in rapid progression of infections and other complications, and an increased probability of systemic damage [41, 42]. Lengthy waiting times will seriously endanger their life, so the waiting time is shorter than those of other disease types.

Patients with more diagnostic items had shorter waiting times. This result reflects the impact of the severity of the disease on the waiting time, to a certain extent. The more diagnoses, the greater the probability that the disease is severe, and the shorter the waiting time compared to other, single disease, types. The results of this study on disease information are consistent with the hospital's actual practice. During the admission process of the case hospital used in this research, one of the rules is to focus on the type of disease and the severity of the disease, instead of scheduling on the principle of first come, first served. These findings suggest that in future admission management, the hospital should establish a more complete and detailed admission system centered on the type of disease, the severity of the disease, and the characteristics of the subspecialties in clinical departments to reduce the waiting time for critically ill patients.

The limitations and future research of this article can be summarized as follows. (1) The study does not consider the health system organizational model as a factor influencing the waiting times in the tertiary hospital. The coordination of primary care, hospitals, and communities improves early identification of health needs, healthcare service provision, and appropriateness [43, 44], reducing waiting times in hospitals and patient's satisfaction. (2) Further research is necessary to demonstrate that the indicators used are useful for the reorganization of services to reduce waiting times. In particular, it is necessary for healthcare professionals to improve the admission process based on the conclusions of this study to help further understand the factors that affect hospital admissions, such as disease care pathway, severity of disease, and services available in the territory [45–47]. (3) Taking into account the actual needs of the hospital, we will classify the waiting times and apply cutting-edge classification algorithms from the field of machine learning to accurately predict waiting times. Combining artificial intelligence technology with the needs of hospital admission will assist in hospitalization management and improve work efficiency.

## 5. Conclusions

The quality of medical service has become the core of hospital management, and continuous customer satisfaction should be the standard. The waiting time of patients in hospital is an important indicator and strongly affects patient satisfaction. In response to the need to reduce patient waiting time, we analyzed the status quo and found that although the average waiting time for admission in the Nephrology Department was less than one week, the standard deviation was large, indicating that the waiting time of patients at the individual level varies considerably, and there is still significant room for improvement.

It is important to find the key factors affecting waiting time for admission, to improve the status quo. Using a review of the literature, combined with interviews and clinical experience, we made full use of the historical data from the hospital, to identify the real problems reflected in the data, using data analysis. We constructed a general linear regression model and analyzed the factors that affected patients' waiting time for admission. The factors found in this study that have a significant impact on waiting time were gender (male), WAIC (Saturday and Sunday), APA (afternoon), RI, and DP (after renal transplant) and NDD (level 4).

The results of this research allow us to develop recommendations for hospital admission management, which can assist in patient management and improve work efficiency. We combined research interviews and literature analysis to provide suggestions for optimizing patients' admission times. These strategies can also reduce the psychological burden on patients.

## Figures and Tables

**Figure 1:** Flow chart of the elective patient admission process.

**Figure 2:** Characteristics of descriptive information. (a) Distribution of gender. (b) The number of cases by age and waiting time in days by age.

**Figure 3:** Characteristics of time-related information. (a) Pie chart of the applied period for admission. (b) Day of issuance of the admission card and waiting time by day.

**Figure 4:** Characteristics of disease-related information. (a) Type of disease and waiting time. (b) The number of disease diagnoses and waiting time.

**Figure 5:** Primary important variable in the linear regression model.

**Table 1:** Variable assignment table.

Categories	Variables	Assignment
Descriptive statistics	Age	1 = juvenile (0–17 years old), 2 = youth (18–40 years old), 3 = middle age (41–65 years old), 4 = old age (over 66 years old)
	Gender	1 = male, 2 = female
Time information	Week of issuing the admission card (WIAC)	1 = Monday, 2 = Tuesday, 3 = Wednesday, 4 = Thursday, 5 = Friday, 6 = Saturday, 7 = Sunday
	Applied period for admission (APA)	1 = morning (00 : 00–11 : 59), 2 = afternoon (12 : 00–23 : 59)
	Registration interval (RI)	Continuous variable
Disease information	Type of disease (TD)	1 = renal biopsy, 2 = peritoneal dialysis, 3 = vascular access, 4 = after renal transplant, 5 = other
	Number of disease diagnosis (NDD)	1 = 1 diagnosis, 2 = 2 diagnoses, 3 = 3 diagnoses, 4 = ≥4 diagnoses

**Table 2:** Comparison of the waiting time of hospitalized patients with different characteristics.

Variable	Cases	Waiting time	*F*	*P*
*Age*			2.365	0.069
Juvenile (0–17 years old)	341	5.08		
Youth (18–40 years old)	4 342	5.39		
Middle age (41–65 years old)	6 234	5.70		
Old age (over 66 years old)	2 419	4.29		

*Gender*			4.705	0.030
Male	7 106	5.72		
Female	6 230	4.88		

*WIAC*			5.648	<0.01
Monday	3 161	4.24		
Tuesday	2 443	4.42		
Wednesday	2 785	6.21		
Thursday	2 524	5.75		
Friday	1 784	5.53		
Saturday	496	9.30		
Sunday	143	3.85		

*APA*			2.365	0.124
Morning	7 530	5.12		
Afternoon	5 806	5.60		

*TD*			2.872	0.021
Renal biopsy	4 408	5.15		
Peritoneal dialysis	1 517	6.97		
Vascular access	3 595	5.31		
After renal transplant	1 492	2.62		
Other	2 324	5.72		

*NDD*			0.083	0.9
1 diagnosis	10 460	5.34		
2 diagnoses	2 190	5.22		
3 diagnoses	444	5.19		
≥4 diagnoses	242	4.96		

**Table 3:** Analysis of linear regression model of the waiting time and factors.

Variables	Unstandardized coefficient		Standardization coefficient	*T*	*P*	95% confidence interval
	*B*	Standard error	*β*			
Intercept	5.647	1.087	0.066	1.353	0.1762	(–0.030, 0.162)
Gender (male)	**0.527**	**0.266**	**0.024**	**1.978**	**0.048**	(0.000, 0.047)
*WIAC*						
Thursday	0.042	0.473	0.002	0.088	0.930	(–0.040, 0.044)
Monday	–0.839	0.453	–0.038	–1.853	0.064	(–0.078, 0.002)
**Sunday**	**–4.244**	**1.328**	**–0.191**	**–3.195**	**0.001**	(–0.309, –0.074)
**Saturday**	**1.704**	**0.777**	**0.077**	**2.194**	**0.028**	(0.008, 0.146)
Wednesday	0.136	0.463	0.006	0.294	0.769	(–0.035, 0.047)
Tuesday	–0.777	0.476	–0.035	–1.633	0.103	(–0.077, 0.007)
APA (Afternoon)	**1.057**	**0.268**	**0.048**	**3.941**	**0.000**	(0.024, 0.071)
**RI**	**0.789**	**0.007**	**0.724**	**121.349**	**0.000**	(0.712, 0.736)

*TD*						
**Renal biopsy**	**–3.091**	**0.741**	**–0.139**	**–4.172**	**0.000**	(–0.205, –0.074)
Peritoneal dialysis	–0.520	0.351	–0.023	–1.481	0.139	(–0.054, 0.008)
Vascular access	–0.373	0.350	–0.017	–1.066	0.286	(–0.048, 0.014)
After renal transplant	1.212	0.722	0.055	1.679	0.093	(–0.009, 0.119)

*NDD*						
2 diagnoses	–1.445	0.993	–0.065	–1.455	0.146	(–0.154, 0.022)
3 diagnoses	–1.472	1.22	–0.065	–1.206	0.228	(–0.176, 0.040)
≥4 diagnoses	**–2.156**	**1.035**	**–0.097**	**–2.082**	**0.037**	(–0.190, –0.007)

*Note.* Bold fields indicate statistically significant variables.

**Table 4:** Collinearity diagnosis results of multivariate linear regression model.

Variables	GVIF	VIF
Gender	1.012	1.006
WIAC	1.036	1.003
APA	1.012	1.006
RI	1.002	1.001
TD	1.039	1.004
NDD	1.008	1.001

## Data Availability

The data used to support the findings of this study are restricted by the Admission Service Center of West China Hospital in order to protect patient privacy. Data are available from West China Hospital for researchers who meet the criteria for access to confidential data.
